# A comparative study of single-channel signal processing methods in fetal phonocardiography

**DOI:** 10.1371/journal.pone.0269884

**Published:** 2022-08-19

**Authors:** Katerina Barnova, Radana Kahankova, Rene Jaros, Martina Litschmannova, Radek Martinek

**Affiliations:** 1 Department of Cybernetics and Biomedical Engineering, Faculty of Electrical Engineering and Computer Science, VSB–Technical University of Ostrava, Ostrava, Czechia; 2 Department of Applied Mathematics, Faculty of Electrical Engineering and Computer Science, VSB–Technical University of Ostrava, Ostrava, Czechia; Effat University, SAUDI ARABIA

## Abstract

Fetal phonocardiography is a non-invasive, completely passive and low-cost method based on sensing acoustic signals from the maternal abdomen. However, different types of interference are sensed along with the desired fetal phonocardiography. This study focuses on the comparison of fetal phonocardiography filtering using eight algorithms: Savitzky-Golay filter, finite impulse response filter, adaptive wavelet transform, maximal overlap discrete wavelet transform, variational mode decomposition, empirical mode decomposition, ensemble empirical mode decomposition, and complete ensemble empirical mode decomposition with adaptive noise. The effectiveness of those methods was tested on four types of interference (maternal sounds, movement artifacts, Gaussian noise, and ambient noise) and eleven combinations of these disturbances. The dataset was created using two synthetic records r01 and r02, where the record r02 was loaded with higher levels of interference than the record r01. The evaluation was performed using the objective parameters such as accuracy of the detection of S1 and S2 sounds, signal-to-noise ratio improvement, and mean error of heart interval measurement. According to all parameters, the best results were achieved using the complete ensemble empirical mode decomposition with adaptive noise method with average values of accuracy = 91.53% in the detection of S1 and accuracy = 68.89% in the detection of S2. The average value of signal-to-noise ratio improvement achieved by complete ensemble empirical mode decomposition with adaptive noise method was 9.75 dB and the average value of the mean error of heart interval measurement was 3.27 ms.

## Introduction

Fetal phonocardiography (fPCG) is a method based on sensing the acoustic signals of the fetal heart from the maternal abdomen providing valuable information about the fetal well-being [1]. The fetal heart sounds (fHSs) were first mentioned in 1650, however, were not officially used in the obstetrics until their rediscovery in the 19th century. The auscultation of fHSs was practiced by placing the ear on the abdominal wall of the mother until 1816, when the stethoscope was invented by the French physician Rene Laennec [2]. The stethoscope allowed doctors to regularly check the fetal heart rate (fHR). Later, with the development of science and technology, an electronic stethoscope was invented to listen to fHSs [3].

The acoustic manifestation of the fetal heart activity is caused by the opening and closing of heart valves. Although there are a total of four types of HSs, only two (S1 and S2) are distinguishable in the fPCG signal. The first HS (herein denoted as S1) is generated during systole by closing the mitral and tricuspid valves. The second HS (herein denoted as S2) is generated during the isovolumic relaxation phase of diastole by closing the aortic and pulmonary valves [4, 5]. The S1 is generally longer with greater magnitude and low frequency vibrations compared to the S2. The systolic interval between S1 and S2 sounds is usually shorter than the diastolic interval between S2 and S1 sounds. It is a narrowband non-stationary signal with a frequency range of 15–110 Hz [3, 4]. In addition to fHSs, the fPCG signal is also able to detect cardiac murmurs. Detection of pathological murmurs contributes to the early detection of congenital valve defects, heart defects, and abnormalities [6, 7]. Pathological murmurs are caused by tissue vibrations or when the laminar blood flow changes to turbulent [8]. It can be classified as systolic (including, for example, aortic valve stenosis, stenosis of bicuspid aortic valve or hypertrophic obstructive cardiomyopathy) and diastolic (including, for example, aortic valve regurgitation, mitral stenosis, or pulmonary valve regurgitation) [6, 8, 9].

The fPCG method has received increasing attention in recent years mainly because it provides more information on cardiac abnormalities and pathologies than cardiotocography (CTG), which is the most common method of the fetal surveillance in today’s clinical practice [4]. In addition, it is a completely passive method, where neither the mother nor the fetus is exposed to any type of radiation, as is the case with CTG [10]. Due to its non-invasiveness, simplicity, and low cost, the fPCG method could become an alternative to CTG suitable for long-term measurement and could also become a technique used for remote home monitoring [11, 12]. The disadvantage of the method is the sensitivity to a wide range of noise, which needs to be filtered in order to obtain clinically valuable information. Moreover, to obtain high quality signal, the measuring probe needs to be placed as close to fetal body as possible, otherwise it is prone to acquiring the unwanted signals instead of the fHS. It is therefore highly dependent on the examiner’s skills.

The most common kind of interference that is sensed along with the useful signal is *ambient noise* caused, for example, by speech, coughing, and other noise produced by the environment. It is a broadband interference comprising frequencies from 10 Hz manifested by a change in the mean value and variation of fPCG [3, 13]. Another type of disturbance that degrades the useful signal is called *motion artifacts* and it is produced either by the maternal body or the fetal one. Such interfering signals associated with the fetus are caused by movement of its limbs, head or change in the fetal position. It is characterized by the frequency range 0–25 Hz and in the time domain it manifests as random impulses. Artifacts caused by maternal movements also manifest as random impulses in fPCG, but in the frequency range 0–100 Hz creating reverberation noise [3, 14]. *Maternal heart sounds* (mHSs) occurring in the 10–40 Hz frequency band can also be considered an interfering signal [3, 15]. Furthermore, the useful signal may be impaired by *uterine contractions*, the intensity and duration of which are affected by the week of pregnancy, which usually occurs in the frequency range 0.2–0.5 Hz. Moreover, *maternal respiratory artifacts* that cause baseline wander and fHR variations also occur in the same frequency range. *Digestive sounds* can also act as disturbances, but not much information has been published about their effect on fPCG. Uterine contractions, respiratory artifacts, digestive sounds or quantization noise of the transducer can be represented as white *Gaussian noise* [3]. To remove these interfering signals and thus extract a high-quality signal providing clinically valuable information, it is necessary to choose a suitable filtering algorithm.

The aim of this study is to compare the performance of eight algorithms: Savitzky-Golay (S-G) filter, finite impulse response (FIR) filter, adaptive wavelet transform (AWT), maximal overlap discrete wavelet transform (MODWT), variational mode decomposition (VMD), empirical mode decomposition (EMD), ensemble empirical mode decomposition (EEMD), complete ensemble empirical mode decomposition with adaptive noise (CEEMDAN). It is important to note that some of the algorithms (e.g. MODWT or CEEMDAN) have not yet been tested and published for the fPCG extraction. Moreover, the effectiveness of these methods in filtering different types of interference was objectively evaluated using several metrics (e.g. accuracy of S1 and S2 detection, SNR improvement and $\bar{|\Delta T_{i}|}$ parameter). The interferences tested included, for example, mHSs, movement artifacts, Gaussian noise, ambient noise, and eleven combinations of these disturbances to best simulate the states that occur in clinical practice. The use of a relatively large number of algorithms, noise scenarios, and evaluation metrics make this study unique and comprehensive. In particular, the evaluation of the accuracy of S2 detection, which is a clinically valuable feature, is quite rare except for very few studies focus on this topic, e.g. [16–18].

## State-of-the-Art

Many authors [3, 13, 15, 19–22] have looked into the design and testing of algorithms for fPCG filtration. As well as the filtering itself, some studies [3, 5, 15, 23, 24] were aimed at detecting S1 sounds, and only a few authors [17, 18] looked into detecting S1 and S2 sounds. The ideal extraction algorithm should both suppress disruptive signals and preserve fPCG morphology so that clinically important information is not lost. A summary of the fPCG signal processing methods will be provided in this section and in Table 1.

- Wavelet transform (WT) was proposed for extraction of fPCG in [13]. The authors did not deal with detection of fHSs, but evaluated the effectiveness of the method only according to signal-to-noise ratio (SNR). The method was tested on 37 synthetic signals, and the best results were achieved with wavelet *coif4* and seven levels of decomposition.
- A comparison study of the WT method was carried out by the authors in [15]. A total of 18 WT-based filters were tested for fPCG extraction. S1 sounds were automatically detected by a PCG-Delineator, which is the threshold-based application. The filters were tested on 37 synthetic records and 119 real ones. Evaluation was based on the accuracy of determining fHR and SNR. And the best results were achieved using wavelet *coif4*, and universal soft thresholding.
- The WT method was also tested in [19]. The authors proposed a new wavelet basis function, designed especially for filtering of fPCG. Fetal wavelet basis function with the threshold rigrsure achieved better results based on mean squared error (MSE) than classic wavelets *db5*, *coif4* and *sym7* with higher convergence speeds.
- The authors in [18] used adaptive WT (AWT) for filtering of fPCG. The most effective filtering was achieved with wavelet *coif2* and six levels of decomposition. Identification of S1 and S2 was based on time intervals between the peaks and their correspondence to physiological values. The method was tested on 14 women between the 36th and 40th week of pregnancy. Evaluation of the perormance of the method was carried out by comparing fHR plots with Doppler ultrasound monitor, and accuracy of 94–97.5% was achieved.
- In [23] a bandpass filter (BPF) with a frequency band of 25–100 Hz was used. For detection of S1 sounds autocorrelation was used as the dominant method, which proved to be very effective for sections with a low level of interference. If, however, this method was not sufficiently precise for sections with higher levels of interference, a further two methods were used for these sections: WT and matching pursuit (MP). The method was tested on 25 real recordings sensed from the abdominal area of pregnant women in the 34th week of pregnancy. This combined approach achieved accuracy in detection of S1 sounds from 92.9% to 98.5%.
- The authors of study [17] created an iterative algorithm combining the WT method and fractal dimension (FD). The WT method was used for removing disturbances from the fPCG signal using wavelet *db4*. The FD method was used for detection of all fHSs. Finally, differentiation between S1 and S2 sounds was carried out, based on the fact that diastolic duration is longer than systolic duration. During testing on 19 synthetic recordings, overall accuracy in detection of fHSs of 89% was achieved.
- AWT methods, empirical mode decomposition (EMD) and ensemble empirical mode decomposition (EEMD) were presented in [3] for fPCG filtration. The Pan-Tompkins algorithm was used for detection of S1 sounds. The method was tested on 12 synthetic recordings, which were distorted by three types of disturbances (ambient noise, Gaussian noise and movement artifacts of the mother and the fetus). Evaluation of the effectiveness of the method was carried out using SNR improvement, mean error of heart interval measurement, fHR, and evaluation of detection of S1 sounds was carried out using statistical parameters: accuracy (ACC), sensitivity (SE), positive predictive value (PPV), and harmonic mean between SE and PPV (F1). According to the ACC parameter, the best results were achieved with AWT in a range of 97.37–100%.
- A single-channel independent component analysis (SCICA) was tested in [20]. First, an appropriate matrix of delays was created, then a multiple FastICA was applied. The method was tested on three real recordings, and the gestation age of the fetuses was 36–40 weeks. The authors did not present any statistical results, but they observed that after filtering of the signals using the given method, S1 and S2 sounds were clearly identifiable.
- Filtering of disturbances with an eigen filter based subspace separation technique with a Wiener filter was presented in [25]. As well as extraction of the fPCG signal the authors also looked into detection of abnormalities (mitral stenosis). An eigenvector based subspace matching system was used for detection of abnormalities. Synthetically generated mitral stenosis was successfully identified with the help of the designed algorithm.
- A single-channel method combining the EMD method, singular value decomposition (SVD) and an efficient version of ICA (EFICA) was proposed in [21]. A combination of all methods was tested on real recordings and even led to effective extraction of signals burdened with high levels of interference. Although the authors did not publish statistical results, they observed that S1 and S2 sounds could clearly be identified.
- The authors in [26] used BPF with a frequency band of 20–200 Hz for filtering of fPCG. Spectograms were then created with the help of short-time Fourier transform (STFT). Finally, the non-negative matrix factorization (NMF) method was used for analysis of the signal and determination of fHR. The authors used real recordings from women in the 38th and 39th week of pregnancy. In addition to fPCG signals, CTG recordings were also made, which served as a reference. The effectiveness of the method was evaluated according to its accuracy in determining fHR with regard to the reference, and accuracy of 84–91% was achieved.
- In [27] a combination of the EMD and and lifting wavelet transform (LWT) methods was used for eliminating interference in the fPCG signal. Subsequently a spectrum of the signal envelope was obtained using Hilbert transform (HT), and the resulting fHR values were obtained using the cepstrum method. The method was tested on 20 real recordings obtained from women between the 30th and 40th week of pregnancy. The authors did not publish statistical results- they only observed that the determined fHR value was accurate.
- The authors in [5] used BPF with a frequency band of 34–54 Hz for filtering of fPCG. Non-linear time Teager energy operator, which identified high-energy peaks and enhanced S1 sounds, was then applied. Finally, a logic block based on amplitude thresholding was used for detection of S1 sounds. During testing on synthetic data, accuracy of 68-99% was achieved in detection of fHR according to ACC parameters.
- In [22] a single-channel method for extraction of fPCG combining EMD, NMF and clustering methods was proposed. The method was tested on 50 real recordings and simultaneously measured CTG was used as a reference. Accuracy of the algorithm in determining fHR was in relation to the reference 83-100%.
- The device for monitoring fHR proposed in [28] used a BPF FIR filter with an order of 124 and a matched filter for filtering of fPCG signals. For determining fHR, a Teager energy operator was applied, which enhanced the positions with fetal heart beats. Finally, autocorrelation was used, which served to detect periodical components and determine fHR. The method was tested on 12 real recordings. The authors did not publish statistical results, but they concluded that this method is effective for determining fHR.
- For filtering of fPCG signals in [24] a combination of matched filter and BPF with a frequency range of 34–54 Hz was used. S1 sounds were then enhanced using a Teager energy operator and detected with the help of autocorrelation and amplitude thresholding. The method was tested on real recordings obtained from women between the 30th and 40th week of pregnancy. The accuracy of the method was evaluated based on determining fHR with regard to reference values of fHR obtained from CTG, which was recorded together with fPCG. The authors concluded that fHR values determined using this method were very close to the reference values determined from CTG.

**Table 1:** Comparison of the fPCG extraction methods.

Author, source	Noise removal	Feature extraction	Results
Sbrollini et al. [13]	WT	–	The best results were obtained with *coif4* and 7 levels of decomposition
Tomassini et al. [15]	WT	S1 detection was performed using threshold-based application (PCG-Delineator)	The best results were obtained with *coif4*, and universal soft thresholding
Chourasia et al. [19]	WT	–	The best results were obtained with new ‘fetal’ avelet basis function
Vaisman et al. [18]	AWT	S1 and S2 identification was based on time intervals between the peaks and their correspondence to physiological values	The best results were obtained with *coif4* and 7 levels of decomposition Accuracy in determining the fHR was 94–97.5%
Kovacs et al. [23]	BPF	S1 detection was based on combination of autocorrelation, WT and MP	The optimal BPF filter Hz band was 25–100 Accuracy in S1 detection was 92.9-98.5%
Koutsiana et al. [17]	WT	fHSs detection was based on FD and S1 and S2 identification was based on physiological values of cardiac cycle	The best results were obtained with *db4* Accuracy in S1 and S2 detection and identification was 89%
Martinek et al. [3]	EMD EEMD AWT	S1 detection was based on Pan-Tompkins algorithm	Accuracy in S1 detection according to ACC was: 46.55-100% 89.02-100% 97.37-100%
Jimenez-Gonzalez et al. [20]	SCICA	–	S1 and S2 were clearly identifiable
Soysa et al. [25]	Eigen filter based subspace separation technique and Wiener filter	Abnormalities detection using an eigenvectorbased subspace matching system	Mitral stenosis was successfully identified
Warbhe et al. [21]	EMD-SVD-EFICA	–	S1 and S2 were clearly identifiable
Dia et al. [26]	BPF	A combination of STFT and NMF was used to determine fHR	The optimal BPF filter band was 20–200 Hz Accuracy in determining the fHR was 84–91%
Huimin et al. [27]	EMD-LWT	A combination of HT and cepstrum was used to determine fHR	The fHR determination was accurate
Cesarelli et al. [5]	BPF	S1 detection was performed using Teager energy operator and logic block based on amplitude thresholding	The optimal BPF filter band was 34–54 Hz Accuracy in determining the fHR was 68–99%
Samieinasab et al. [22]	EMD-NMF-Clustering	–	Accuracy in determining the fHR was 83–100%
Zahorian et al. [28]	FIR-Matched filter	A combination of Teager energy operator and autocorrelation was used to determine fHR	The fHR determination was accurate
Ruffo et al. [24]	BPF-Matched filter	S1 detection was performed using Teager energy, autocorrelation and amplitude thresholding	The fHR values were very close to the reference values

From the above it emerges that objective comparison of testing method performance is problematic, because authors use different signals (real or synthetic) disturbed by various levels and types of interference. Some authors [3, 5, 17, 18, 22, 23, 26] then evaluate the effectiveness of filtering using objective statistical parameters and some [20, 21, 27] only subjectively evaluate the extracted waveform. The aim of this study is to carry out an objective and uniform comparison of eight algorithms for filtering of fPCG for various types and levels of disturbance and evaluate their effectiveness using statistical parameters. This comparative study could therefore help find the optimal algorithm for processing fPCG, which could be implemented in devices for home monitoring and analysis of the heart activity of fetuses.

## Materials and methods

On the basis of in-depth research eight algorithms (S-G filter, FIR filter, AWT, MODWT, VMD, EMD, EEMD, and CEEMDAN) were chosen for filtering fPCG which have the potential to effectively filter interference. This section also includes a description of the reference signals and disturbances which were generated for testing these algorithms. The evaluation parameters which were used for evaluating the quality of filtering and accuracy of detection of S1 and S2 sounds are also described.

### Filtration algorithms

This subsection summarises the basic information about algorithms. As the majority of the algorithms are very well described in the literature, only the basic facts are given here. For each method the literature is cited, where extra information can be found.

- *Savitzky-Golay filter*—polynomial S-G filter is a widely used method for smoothing and differentiating time series, and also biomedical data [29]. The technique is based on least squares fitting of a lower order polynomial to a number of consecutive points [30]. The aim of filtering using S-G is to find co-efficients that increase the accuracy of data, and also maintain the trend of the given signal [29]. To achieve good results, it is necessary to find a compromise when choosing the length of the window and the polynomial order for the tested data. A detailed description of this technique can be obtained in [29–31]. S-G was used in [32] as part of the filtering algorithm for fPCG and for processing of adult PCG in [33, 34].
- *Finite impulse response filter*—the non-recursive FIR filter can also be categorised as one of the frequently used filters for processing biomedical signals [35]. This is a filter whose impulse response has finite length. The advantage of the filter is its stability and linear phase response, where there is the same delay in harmonic sections with no phase distortion [35]. For correct functioning of the FIR filter it is necessary to choose an appropriate filter length and cut-off frequency. Further information can be found in [31, 35, 36]. The FIR filter was tested for filtering of fPCG in [28] and for filtering of adult PCG in [37].
- *Adaptive wavelet transform*—methods based on WT are among the most frequently used techniques for processing non-stationary signals, and thus also for filtering of fPCG. The advantage of the method is the representation of the processed signal both in a time and frequency domain [3, 19]. The first step is the decomposition of the input signal, when co-efficients are obtained. In the case of AWT, this is followed by adaptive thresholding of these co-efficients. Each co-efficient is assigned a certain threshold value, which corresponds to the changes in interference output in the signal (this is achieved using a moving window) [3]. Inverse WT is applied for reconstruction of the filtered signal. In order for filtering of the signal to be effective, the appropriate type and width of wavelet, and the appropriate number of decomposition levels must be chosen. More information about the method can be found in [38]. WT was tested for the purposes of fPCG filtering in [13, 15, 19], and speciically the AWT method in [3, 18].
- *Maximal overlap discrete wavelet transform*—the MODWT method can also be placed in the WT family (also known as undecimated discrete wavelet transform), which is based on the principle of leaving out the down-sampling process [39]. The wavelet co-efficients therefore have the same length as the input signal at each level, and offer better approximisation. Inverse WT and thresholding follow [40]. Again the choice of the type of wavelet, wavelet length, and the number of decomposition levels for the given type of signal play an important role. Further information can be obtained in [39, 40]. For processing adult PCG signals the method in [41] was used.
- *Variational mode decomposition*—the VMD method is a relatively new quasi-orthogonal technique based on the decomposition of the input signal into intrinsic mode functions (IMFs). These IMFs represent a separated frequency band of the processed signal [42, 43]. The method uses a calculation of a one-way frequency spectrum using HT and the shift of individual modes to baseband. The width of the band of each mode is estimated using Dirichlet energy of the demodulated signal [44]. VMD is an alternative to the EMD method, however in contrast to EMD individual IMFs are extracted simultaneously and non-recursively [42]. More detailed information can be found in [42–44]. For the purposes of processing fPCG the method in [45] was used, and for processing adult PCG the method in [44] was introduced.
- *Empirical mode decomposition*—EMD is a filtering technique appropriate for processing non-stationary and non-linear signals. As in the VMD method, the input signal is decomposed into internal oscillatory functions—IMFs, which represent a specific frequency band [21]. The principle of the method is based on the detection of upper and lower envelope of the signal by detecting the local maxima and minima. The mean of envelopes is then calculated and subtracted from the input signal. The resulting signal is denoted as IMF1 if it fulfills the conditions for IMFs. Further IMFs are extracted by repeating the whole procedure, however instead of the input signal, residue is used, which is created by subtracting IMF1 from the input signal [21, 46, 47]. The effectiveness of the EMD method is lowered by the *mode mixing* problem, where one IMF covers multiple components with different frequencies [48]. Further information can be obtained in [3, 21, 46–48]. The method was tested for processing fPCG in [3, 21, 22, 27] and for processing adult PCG in [49, 50].
- *Ensemble empirical mode decomposition*—the EEMD method was proposed in order to overcome the limitations of the EMD method, and resulted in more effective filtering of signals. EEMD works on the principle of adding white noise to the input signal and carrying out a pre-chosen number of EMD cycles [3, 51]. Individual IMFs, which are created by averaging the results of all EMD cycles, are the output of the algorithm [3, 52]. The disadvantage of the EEMD method is its low computational speed. A detailed description is presented in [3, 51, 52]. The EEMD method was used for processing fPCG in [3], and for processing adult PCG in [53, 54].
- *Complete ensemble empirical mode decomposition with adaptive noise*—the CEEMDAN method was designed with the aim of overcoming the limitations of the EEMD method. CEEMDAN works on the same principle as EEMD with small differences [55]. Paired positive and negative adaptive white noise is added to the input signal, which is able to contribute more to elimination of *mode mixing*. The predetermined number of EMD cycles is then carried out and the resulting IMFs are determined by averaging the outputs of all EMD cycles [55, 56]. The resulting IMFs are however counted sequentially, which leads to an increase in the computational speed of the algorithm. More information about the method can be found in [55, 56]. Processing of adult PCG using CEEMDAN was carried out in [54, 57].

### Fetal heart sounds detection

Detection of S1 and S2 sounds was inspired by study [58]. The principle of the method is based on a combination of HT, and threshold and deciding factors. First, the envelope of the input signal was detected using HT. The signal envelope contained residues of interference, so it was smoothed out using a low-pass filter (LPF). All peaks were then detected, and potential S1 and S2 sounds were found. Peaks which were above the threshold value, which was set as 0.4 times the maximal amplitude of the envelope, were labelled as potential S1 and S2 sounds. Other peaks were excluded.

In order to avoid detection of extra peaks, a principle was established for their elimination, through setting a minimum time interval between peaks of 100 ms. If the time interval was shorter, an extra peak was searched for between peaks. If more such peaks were found in this interval, the peak with the highest amplitude was preserved, and lower peaks were excluded.

Due to the variability of fHSs amplitude, it was also necessary to deal with the possibility that some of the fHSs appeared under the set threshold and could therefore affect subsequent classification. After excluding extra peaks, the shortest interval between two fHSs was chosen and a limit with a value twice as large as that interval was defined. If a time interval with a value larger than the assigned limit was then detected, the peak with the maximum amplitude in that interval was found and the lost peak was restored.

Finally, peaks classified as S1 and S2 sounds were detected on the basis of the physiological characteristics of the heartbeat. The systolic interval between S1 and S2 sounds is usually shorter than the disastolic interval between S1 and S2 sounds. The longest time interval was discovered between the detected peaks, and the first peak was labelled as S2 and the second as S1. Further peaks were labelled in sequence. An example of individual detection steps is shown in Fig 1.

**Fig 1:** S1 and S2 sounds detection procedure: a) input signal, b) envelope detection using HT, c) detected signal envelope with interference residues, d) smoothed envelope using LPF, e) detection of fHSs above the threshold value (the blue line indicates the threshold value), and f) resulting classification of S1 and S2 sounds.

### Reference signals and noise

For testing filtering methods, it was necessary to choose appropriate signals. Unfortunately at the current time there are only three publicly accessible databases: *Shiraz University Fetal Heart Sounds Database* [22], *Fetal PCGs Database available* in *PhysioBank* archive [59], both containing real data. A *Simulated Fetal Phonocardiograms Database* [5] containing synthetically generated signals with different fetal states (physiological or pathological) and recording conditions. One obstacle in testing algorithms on real recordings is the absence of a reference signal against which the accuracy of filtering methods could be evaluated.

For this reason, we used our own synthetic signals for testing. We generated two reference signals (r01 a r02), to which we added the four most commonly occurring types of disturbances during fPCG recording in real conditions (mHSs, maternal and fetal movement artifacts, white Gaussian noise and ambient noise). In order to best simulate the influence of disturbances on the quality of the signal in real conditions, where multiple types of interference can work simultaneously, we additionally loaded the reference signals with combinations of individual types of disturbance (e.g. mHSs and movement artifacts, Gaussian noise and ambient noise etc.). In total for each signal 15 types of disturbances were tested (four individual types of disturbance and eleven combined types). Signal r01 was loaded with lower levels of disturbance (SNR of signal with mHSs: -0.53 dB, movement artifacts: -0.84 dB, Gaussian noise: -1.20 dB, and ambient noise: -2.25 dB), while signal r02 was loaded with lower levels of disturbance (SNR of signal with mHSs: -1.82 dB, movement artifacts: -2.49 dB, Gaussian noise: -3.56 dB, and ambient noise: -5.74 dB). The SNR values of input disturbed signals can be found in Tables 2–7. An example of reference signals and individual types of disturbance can be seen in Fig 2. All used input signals (with and without interference) can be found at *figshare data repository* [60] along with all extracted signals that were obtained using the tested algorithms.

**Fig 2:** An example of reference signals and four individual types of disturbance which the reference signals were loaded with. Example a) represents reference signal r01 and a lower level of disturbance compared to b) reference signal r02, which was loaded with higher levels of disturbance (SNR values of input disturbance signals are in Tables 2–7).

**Table 2:** Setting parameters for S-G filter, FIR filter, AWT, and MODWT.

Type of interference	Record	SNR of signal with noise (dB)	Algorithms						
			S-G		FIR	AWT		MODWT	
			Window	Polynomial	Filter	Wavelet	Decomp.	Wavelet	Decomp.
			length	order	order	type	level	type	level
mHSs	r01	-0.53	20	7	31	*sym4*	3	*db5*	4
	r02	-1.82	40	10	90	*sym6*	3	*db4*	4
Movement artifacts	r01	-0.84	26	9	16	*coif5*	3	*sym3*	4
	r02	-2.49	34	7	150	*db4*	3	*coif5*	4
Gaussian noise	r01	-1.20	12	10	2	*coif5*	3	*db4*	4
	r02	-3.56	16	6	5	*coif5*	3	*sym3*	4
Ambient noise	r01	-2.25	16	10	3	*coif5*	3	*coif4*	4
	r02	-5.74	32	8	10	*coif5*	3	*db5*	4
mHSs, Movement artifacts	r01	-1.45	36	6	105	*sym6*	3	*coif4*	4
	r02	-3.61	26	4	142	*sym6*	3	*coif5*	4
mHSs, Gaussian noise	r01	-1.60	12	8	60	*db5*	3	*coif4*	4
	r02	-4.48	32	8	92	*coif5*	3	*coif5*	4
mHSs, Ambient noise	r01	-2.57	30	8	138	*coif5*	3	*sym3*	4
	r02	-6.30	28	6	114	*coif5*	3	*db5*	4
Movement artifacts, Gaussian noise	r01	-2.65	52	10	97	*db6*	3	*sym6*	4
	r02	-5.94	52	9	136	*sym4*	3	*coif5*	4
Movement artifacts, Ambient noise	r01	-3.52	26	4	88	*coif5*	3	*coif5*	4
	r02	-7.43	58	8	111	*db3*	3	*sym5*	4
Gaussian noise, Ambient noise	r01	-4.65	22	6	16	*coif4*	3	*db6*	4
	r02	-9.43	44	6	10	*db5*	3	*coif5*	4
mHSs, Movement artifacts, Gaussian noise	r01	-2.94	36	6	84	*db6*	3	*sym5*	4
	r02	-6.48	58	8	133	*sym6*	3	*sym6*	4
mHSs, Movement artifacts, Ambient noise	r01	-3.75	40	6	98	*coif4*	3	*coif5*	4
	r02	-7.82	50	6	210	*coif5*	3	*coif4*	4
mHSs, Gaussian noise, Ambient noise	r01	-4.84	48	10	58	*coif5*	3	*coif5*	4
	r02	-9.67	32	4	158	*sym6*	3	*sym6*	4
Movement artifacts, Gaussian noise, Ambient noise	r01	-5.73	32	4	96	*db5*	3	*coif3*	4
	r02	-10.57	50	6	6	*sym5*	3	*db5*	4
mHSs, Movement artifacts, Gaussian noise, Ambient noise	r01	-5.87	40	6	107	*sym6*	3	*coif3*	4
	r02	-10.76	50	6	9	*db3*	3	*db5*	4

**Table 3:** Setting parameters for VMD, EMD, EEMD and CEEMDAN.

Type of interference	Record	SNR of signal with noise (dB)	Algorithms							
			VMD	EMD	EEMD			CEEMDAN		
			IMF	IMF	N	Nstd	IMF	N	Nstd	IMF
mHSs	r01	-0.53	2+3	2+3+4	50	0.8	4	10	0.7	2+3
	r02	-1.82	2+3	2+4+6	10	0.6	3+4	50	0.2	2
Movement artifacts	r01	-0.84	1+2+3	2	10	0.4	3+4	10	0.3	2+3
	r02	-2.49	2+3	2+5	10	0.6	2+4+6	30	0.7	2+3
Gaussian noise	r01	-1.20	1+2+3	3+4+5	30	0.1	3+4	10	0.4	2+3
	r02	-3.56	1+2+3	3+4+5	10	0.3	4+5	10	0.5	2+3
Ambient noise	r01	-2.25	1+2+3	3+4+5	10	0.1	3+4+5	10	0.6	2+3
	r02	-5.74	1+2+3	3+4+5	30	0.9	4+5	50	0.6	2+3+4
mHSs, Movement artifacts	r01	-1.45	2+3	2	10	0.2	3+4	50	0.2	2
	r02	-3.61	2+3	2+5	50	0.7	2+5	50	0.8	3
mHSs, Gaussian noise	r01	-1.60	1+2+3	3+4	30	0.1	3+4	10	0.5	2+3
	r02	-4.48	1+2+3	4	30	0.4	2+4	50	0.7	2+3
mHSs, Ambient noise	r01	-2.57	1+2+3	3+4	30	0.6	4+5	30	0.5	2+3
	r02	-6.30	1+2+3	3+4+5	50	0.7	4+5	30	0.8	3+5+6
Movement artifacts, Gaussian noise	r01	-2.65	1+2	2+3+4	50	0.6	4	10	0.7	2+3+6
	r02	-5.94	1+2	3+4	50	0.3	4	30	0.8	3
Movement artifacts, Ambient noise	r01	-3.52	1+2	3+4	50	0.3	2+4	30	0.6	2+3
	r02	-7.43	1+3	2+4+5	30	0.5	4+5	50	0.9	3
Gaussian noise, Ambient noise	r01	-4.65	1+2+3	3+4+5	50	0.9	4+5	50	0.6	2+3+5
	r02	-9.43	1	2+4+5	50	0.8	2+3+5	50	0.7	3
mHSs, Movement artifacts, Gaussian noise	r01	-2.94	1+2	2+3+4	50	0.7	4	30	0.5	2+3+5
	r02	-6.48	2+3	4	50	0.4	4	10	0.8	3+6
mHSs, Movement artifacts, Ambient noise	r01	-3.75	1+2	3+4	50	0.4	4	30	0.5	2+3+6
	r02	-7.82	1+2	2+4+5	50	0.3	4+5	30	0.8	3
mHSs, Gaussian noise, Ambient noise	r01	-4.84	1+2+3	4+5	50	0.4	4+5	50	0.5	2+3
	r02	-9.67	1+2	2+3+4+5	50	0.9	2+3+5	10	0.9	3
Movement artifacts, Gaussian noise, Ambient noise	r01	-5.73	1+2	4+5	30	0.3	4+5	30	0.8	3
	r02	-10.57	1	4+5	50	0.8	2+3+5	10	0.7	3
mHSs, Movement artifacts, Gaussian noise, Ambient noise	r01	-5.87	1+2	4+5	50	0.7	4+5	50	0.8	3+6
	r02	-10.76	1	4+5	30	0.8	2+3+5	30	0.9	3

**Table 4:** Statistical evaluation of the accuracy according to ACC (%) of S1 sounds detection.

Type of interference	Record	SNR of signal with noise (dB)	Algorithms							
			S-G	FIR	AWT	MODWT	VMD	EMD	EEMD	CEEMDAN
mHSs	r01	-0.53	**100.00**	**100.00**	**100.00**	**100.00**	88.58	**100.00**	**100.00**	**100.00**
	r02	-1.82	93.52	97.30	93.39	98.14	86.14	96.35	**100.00**	99.13
Movement artifacts	r01	-0.84	**100.00**	**100.00**	**100.00**	**100.00**	88.58	**100.00**	**100.00**	**100.00**
	r02	-2.49	93.36	91.21	96.07	93.50	86.26	**96.59**	96.58	95.43
Gaussian noise	r01	-1.20	**100.00**	**100.00**	**100.00**	**100.00**	88.71	**100.00**	**100.00**	**100.00**
	r02	-3.56	**100.00**	**100.00**	**100.00**	**100.00**	87.69	99.71	**100.00**	**100.00**
Ambient noise	r01	-2.25	**100.00**	**100.00**	**100.00**	**100.00**	88.58	**100.00**	**100.00**	**100.00**
	r02	-5.74	98.55	98.99	**99.71**	99.13	87.19	95.72	99.56	97.69
mHSs, Movement artifacts	r01	-1.45	99.57	99.56	98.99	99.85	88.32	99.85	**100.00**	**100.00**
	r02	-3.61	80.67	84.46	85.55	90.08	77.04	92.31	**95.89**	95.53
mHSs, Gaussian noise	r01	-1.60	**100.00**	**100.00**	**100.00**	**100.00**	88.97	**100.00**	**100.00**	**100.00**
	r02	-4.48	90.34	97.02	93.05	98.70	83.66	94.48	98.40	**99.13**
mHSs, Ambient noise	r01	-2.57	**100.00**	**100.00**	**100.00**	**100.00**	88.97	98.69	**100.00**	**100.00**
	r02	-6.30	87.25	92.64	92.93	97.15	83.88	88.72	95.09	**98.00**
Movement artifacts, Gaussian noise	r01	-2.65	97.00	95.04	98.70	97.84	85.14	96.10	**99.85**	97.12
	r02	-5.94	72.39	62.29	71.84	68.73	58.53	62.62	75.28	**76.51**
Movement artifacts, Ambient noise	r01	-3.52	96.04	89.99	97.29	94.83	81.59	87.86	**97.99**	94.23
	r02	-7.43	**72.04**	55.07	66.74	59.20	66.70	60.68	65.49	70.50
Gaussian noise, Ambient noise	r01	-4.65	99.27	98.98	**99.85**	99.56	88.46	98.84	**99.85**	99.71
	r02	-9.43	88.92	72.94	87.13	79.41	75.45	70.20	91.51	**92.49**
mHSs, Movement artifacts, Gaussian noise	r01	-2.94	96.16	92.71	97.58	97.18	83.69	94.69	**98.84**	95.86
	r02	-6.48	70.46	59.05	65.04	66.16	63.90	64.65	70.32	**80.23**
mHSs, Movement artifacts, Ambient noise	r01	-3.75	96.19	89.13	96.74	94.56	80.23	87.45	**98.41**	93.81
	r02	-7.82	65.86	52.18	60.90	60.41	46.74	58.98	61.73	70.58
mHSs, Gaussian noise, Ambient noise	r01	-4.84	98.70	95.83	99.57	99.57	88.72	98.70	**99.71**	98.55
	r02	-9.67	80.12	63.44	76.80	75.24	74.59	65.04	85.22	**89.44**
Movement artifacts, Gaussian noise, Ambient noise	r01	-5.73	90.63	74.13	89.64	82.77	74.57	77.72	84.42	**94.48**
	r02	-10.57	**60.02**	42.03	51.18	50.38	51.38	43.00	55.53	57.41
mHSs, Movement artifacts, Gaussian noise, Ambient noise	r01	-5.87	85.56	72.14	87.04	82.26	71.92	75.66	82.60	**95.13**
	r02	-10.76	53.46	41.51	47.87	48.76	50.24	42.90	52.41	**55.02**
Average values	–	–	88.87	83.92	88.45	87.78	78.48	84.92	90.16	**91.53**

**Table 5:** Statistical evaluation of the accuracy according to ACC (%) of S2 sounds detection.

Type of interference	Record	SNR of signal with noise (dB)	Algorithms							
			S-G	FIR	AWT	MODWT	VMD	EMD	EEMD	CEEMDAN
mHSs	r01	-0.53	87.32	**100.00**	86.45	**100.00**	88.57	87.19	95.15	**100.00**
	r02	-1.82	59.04	90.33	58.35	89.51	80.03	55.36	**94.42**	92.89
Movement artifacts	r01	-0.84	98.55	**98.84**	84.25	94.98	85.71	96.55	95.56	98.41
	r02	-2.49	59.02	72.84	48.71	73.40	72.16	77.63	67.23	**78.28**
Gaussian noise	r01	-1.20	**100.00**	**100.00**	80.00	99.13	44.56	**100.00**	99.71	99.27
	r02	-3.56	**99.13**	98.69	60.81	88.36	55.39	94.77	82.12	94.83
Ambient noise	r01	-2.25	**100.00**	99.71	67.31	94.15	53.96	99.27	99.27	98.70
	r02	-5.74	**90.76**	89.75	54.10	77.12	60.09	41.53	82.18	84.58
mHSs, Movement artifacts	r01	-1.45	72.87	77.14	65.83	89.41	83.54	92.09	93.04	**95.99**
	r02	-3.61	42.05	66.79	32.61	65.83	60.09	**70.17**	50.62	52.34
mHSs, Gaussian noise	r01	-1.60	84.97	**99.71**	62.12	96.26	35.17	98.55	99.27	97.69
	r02	-4.48	56.64	78.64	33.64	**79.21**	19.76	57.71	58.67	75.86
mHSs, Ambient noise	r01	-2.57	83.29	97.12	55.32	95.55	43.64	95.28	93.63	**98.26**
	r02	-6.30	51.09	52.07	32.04	47.13	37.76	44.86	**61.66**	40.79
Movement artifacts, Gaussian noise	r01	-2.65	76.53	89.10	60.05	84.21	79.95	88.89	71.26	**89.89**
	r02	-5.94	27.42	42.42	28.89	39.78	31.71	43.32	**44.09**	36.98
Movement artifacts, Gaussian noise	r01	-3.52	67.31	**82.92**	59.93	77.68	71.98	77.68	78.71	81.20
	r02	-7.43	24.50	30.59	28.99	**39.15**	20.77	26.76	37.81	36.98
Gaussian noise, Ambient noise	r01	-4.65	95.42	**96.28**	61.09	86.25	68.37	58.13	91.82	93.08
	r02	-9.43	36.16	33.03	**43.96**	37.30	43.49	23.50	19.09	34.02
mHSs, Movement artifacts, Gaussian noise	r01	-2.94	61.16	80.24	49.42	81.22	65.95	**86.47**	73.27	84.32
	r02	-6.48	23.28	35.51	26.88	**46.85**	38.15	38.36	45.21	34.64
mHSs, Movement artifacts, Ambient noise	r01	-3.75	54.80	62.03	50.91	75.73	66.55	77.43	64.31	**80.13**
	r02	-7.82	22.19	33.39	28.41	**37.81**	28.77	26.56	33.83	32.43
mHSs, Gaussian noise, Ambient noise	r01	-4.84	77.76	81.75	54.98	84.23	57.74	76.65	89.23	**90.92**
	r02	-9.67	28.32	38.87	33.30	**41.42**	30.82	23.80	18.67	33.48
Movement artifacts, Gaussian noise, Ambient noise	r01	-5.73	39.07	37.78	43.49	42.15	47.51	48.83	**60.07**	35.36
	r02	-10.57	20.32	23.00	23.31	**28.02**	24.44	24.62	17.82	24.33
mHSs, Movement artifacts, Gaussian noise, Ambient noise	r01	-5.87	41.45	42.12	43.30	45.99	46.08	46.97	**59.26**	41.72
	r02	-10.76	19.88	23.64	21.71	24.80	20.31	21.90	17.97	**29.30**
Average values	–	–	60.01	68.48	49.34	68.75	52.10	63.36	66.50	**68.89**

**Table 6:** Statistical evaluation of the SNR improvement (dB).

Type of interference	Record	SNR of signal with noise (dB)	Algorithms							
			S-G	FIR	AWT	MODWT	VMD	EMD	EEMD	CEEMDAN
mHSs	r01	-0.53	9.29	10.77	9.23	4.04	7.90	9.17	**15.14**	14.45
	r02	-1.82	4.60	10.36	4.59	9.18	8.25	6.77	**13.32**	11.10
Movement artifacts	r01	-0.84	7.57	7.84	7.93	4.07	5.62	10.82	**11.16**	9.82
	r02	-2.49	4.05	6.19	4.28	4.75	5.79	6.46	**7.80**	7.43
Gaussian noise	r01	-1.20	7.83	7.22	**14.10**	3.59	7.27	9.73	10.33	12.07
	r02	-3.56	7.86	7.03	**11.23**	9.20	6.99	6.28	10.83	8.97
Ambient noise	r01	-2.25	7.43	7.37	**13.96**	6.08	7.18	7.60	8.05	10.16
	r02	-5.74	9.75	7.95	**12.27**	7.97	6.92	5.18	10.59	7.99
mHSs, Movement artifacts	r01	-1.45	5.68	8.50	5.73	4.75	6.99	**10.12**	9.47	10.03
	r02	-3.61	2.79	6.14	2.82	3.87	6.49	6.87	**9.58**	8.58
mHSs, Gaussian noise	r01	-1.60	6.87	**11.91**	8.98	5.53	6.84	9.04	10.52	10.82
	r02	-4.48	5.64	9.05	6.04	6.36	5.76	**9.08**	4.91	**9.08**
mHSs, Ambient noise	r01	-2.57	8.78	10.94	9.58	5.88	6.85	7.33	**11.18**	10.07
	r02	-6.30	6.92	8.70	7.62	6.55	6.27	4.60	9.40	**11.60**
Movement artifacts, Gaussian noise	r01	-2.65	5.70	6.95	5.98	2.56	5.47	4.68	**9.82**	7.30
	r02	-5.94	4.39	5.18	4.50	6.16	4.55	4.63	8.28	**9.09**
Movement artifacts, Ambient noise	r01	-3.52	6.49	6.79	6.62	2.98	5.99	5.34	5.23	**6.99**
	r02	-7.43	5.98	5.37	5.97	6.00	6.68	2.20	6.44	**9.79**
Gaussian noise, Ambient noise	r01	-4.65	9.14	9.01	**12.08**	5.38	6.94	5.61	11.06	8.73
	r02	-9.43	11.33	6.83	11.29	8.49	11.32	1.53	1.15	**13.46**
mHSs, Movement artifacts, Gaussian noise	r01	-2.94	5.10	7.07	5.20	3.87	5.25	4.89	**9.91**	6.90
	r02	-6.48	3.68	5.21	3.57	5.55	7.45	6.70	**8.73**	8.43
mHSs, Movement artifacts, Ambient noise	r01	-3.75	5.88	6.71	5.86	3.17	5.71	5.52	**9.41**	6.76
	r02	-7.82	5.15	5.30	4.72	6.67	4.76	2.19	6.06	**9.74**
mHSs, Gaussian noise, Ambient noise	r01	-4.84	9.20	9.58	9.87	4.75	6.78	8.43	**10.34**	8.89
	r02	-9.67	9.02	8.15	8.83	9.95	8.09	0.69	1.34	**12.73**
Movement artifacts, Gaussian noise, Ambient noise	r01	-5.73	7.06	6.54	6.93	4.67	6.49	6.32	7.40	**10.16**
	r02	-10.57	7.12	3.53	6.59	5.54	8.46	5.90	1.91	**10.55**
mHSs, Movement artifacts, Gaussian noise, Ambient noise	r01	-5.87	6.29	6.41	6.31	4.77	6.29	6.15	7.56	**9.90**
	r02	-10.76	6.40	3.31	6.11	5.68	7.94	5.74	1.98	**10.80**
Average values	–	–	6.77	7.40	7.63	5.60	6.78	6.19	8.30	**9.75**

**Table 7:** Statistical evaluation of the parameter $\bar{|\Delta T_{i}|}$ (ms).

Type of interference	Record	SNR of signal with noise (dB)	Algorithms							
			S-G	FIR	AWT	MODWT	VMD	EMD	EEMD	CEEMDAN
mHSs	r01	-0.53	0.21	0.12	0.20	0.10	0.48	0.22	**0.06**	0.12
	r02	-1.82	3.60	1.74	3.67	1.48	1.29	2.15	**0.21**	0.90
Movement artifacts	r01	-0.84	0.23	0.22	0.18	0.31	0.64	**0.15**	0.16	0.26
	r02	-2.49	3.70	3.75	2.70	3.56	3.47	1.91	**1.87**	2.53
Gaussian noise	r01	-1.20	0.03	0.03	**0.01**	0.70	0.52	0.06	0.06	0.06
	r02	-3.56	0.35	0.35	**0.14**	0.39	0.44	0.60	0.27	0.34
Ambient noise	r01	-2.25	0.09	0.11	0.02	**0.12**	0.49	0.16	0.13	0.13
	r02	-5.74	1.36	1.21	**0.61**	1.07	0.91	2.38	0.83	1.28
mHSs, Movement artifacts	r01	-1.45	0.78	0.60	1.14	0.45	0.83	**0.38**	0.56	0.47
	r02	-3.61	7.19	5.88	6.44	4.58	5.39	3.50	**2.01**	2.83
mHSs, Gaussian noise	r01	-1.60	0.26	0.14	0.24	**0.08**	0.62	0.25	0.11	0.22
	r02	-4.48	4.75	2.07	3.91	1.08	2.94	2.14	1.04	**0.99**
mHSs, Ambient noise	r01	-2.57	0.32	**0.18**	0.26	0.25	0.64	0.95	0.25	0.23
	r02	-6.30	5.30	3.51	4.04	1.97	2.90	4.86	2.71	**1.75**
Movement artifacts, Gaussian noise	r01	-2.65	2.02	2.31	1.25	1.57	2.32	2.44	**0.58**	1.66
	r02	-5.94	10.58	11.43	10.22	10.68	11.36	10.30	**7.47**	9.49
Movement artifacts, Ambient noise	r01	-3.52	2.41	4.27	1.74	2.66	3.95	4.06	**1.34**	2.69
	r02	-7.43	10.84	12.88	11.72	12.70	10.45	11.27	11.11	**10.40**
Gaussian noise, Ambient noise	r01	-4.65	0.83	1.01	**0.37**	0.76	0.67	1.15	0.46	0.57
	r02	-9.43	5.70	9.34	5.98	7.89	6.70	9.40	4.56	**3.91**
mHSs, Movement artifacts, Gaussian noise	r01	-2.94	2.09	3.21	1.81	2.00	3.02	2.92	**1.10**	2.51
	r02	-6.48	10.99	12.02	11.28	11.13	10.42	10.80	8.49	**7.33**
mHSs, Movement artifacts, Gaussian noise	r01	-3.75	2.15	4.49	2.11	3.00	4.60	4.44	**1.51**	2.99
	r02	-7.82	11.75	13.24	11.95	12.37	12.75	11.12	11.60	**10.18**
mHSs, Gaussian noise, Ambient noise	r01	-4.84	1.26	2.13	0.69	0.79	0.88	1.15	**0.64**	1.37
	r02	-9.67	8.02	10.91	8.78	8.82	7.53	10.49	6.68	**4.30**
Movement artifacts, Gaussian noise, Ambient noise	r01	-5.73	4.55	8.65	4.60	6.90	6.41	8.23	6.82	**3.25**
	r02	-10.57	12.11	14.93	13.85	13.81	12.73	13.87	12.51	**10.91**
mHSs, Movement artifacts, Gaussian noise, Ambient noise	r01	-5.87	6.29	9.12	5.68	6.90	7.74	8.63	7.03	**2.67**
	r02	-10.76	12.87	13.86	13.75	13.89	12.84	13.30	12.91	**11.87**
Average values	-	-	4.42	5.12	4.31	4.40	4.53	4.78	3.50	**3.27**

Generation of reference signals and individual types of disturbance was inspired by study [4], and can be summarised as follows:

- *Reference signals*—reference signals were modelled using Gaussian modulated sinusoid (detailed information can be found in [4]). Signals with a length of 300 s represented a fetus with a gestational age of 40 weeks, with a sampling frequency of 1000 Hz and average fHR of 140 bpm. The ratio of S1 and S2 sounds was 1.7, central frequency of S1 was 36.89 Hz, central frequency of S2 was 55.18 Hz and S1 and S2 time inter-distance was 140 ms.
- *mHSs*—interference occurs in the frequency band 10–40 Hz and like the reference signals was modelled using Gaussian modulated sinusoid. Average mHR was 70 bpm, the ratio of S1 and S2 sounds was 1.54, central frequency of S1 was 16.93 Hz, central frequency of S2 was 30.44 and S1 and S2 time inter-distance was 331 ms.
- *Maternal and fetal movement artifacts*—artifacts caused by movement of limbs, head, or change in position of the fetus occurring in the frequency band 0–25 Hz and manifesting as random impulses in fPCG. Artifacts caused by movement of the mother also manifested themselves as random impulses in fPCG, though in a frequency range of 0–100 Hz. Interference was modelled as random pulses with a fixed amplitude lasting 0.5 to 1.5 s.
- *White Gaussian noise*—this is random interference, which can be caused by womb contractions, maternal breathing artifacts, digestive sounds or quantization noise of the transducers. Interference was modelled as random Gaussian noise with the same power in any band of the same width.
- *Ambient noise*—broadband interference comprising frequencies from 10 Hz, caused by for instance speech, coughing, closing doors etc. Interference was modelled by a fifth order Butterworth high-pass filter with a cut-off frequency of 100 Hz.

### Evaluation methods

Objective evaluation of the effectiveness of the methods was carried out by comparing the accuracy of detection of S1 and S2 sounds, calculation of SNR improvement and determination of mean error of heart interval measurement $\bar{|\Delta T_{i}|}$.

- *Accuracy of S1 and S2 sounds detection*—in order to establish the accuracy of fHSs detection first of all true positive (TP) values were established, as correctly detected S1 or S2 sounds, set ±50 ms [3, 61] from equivalent S1 or S2 sounds in the reference signal. False positive (FP) values were then set, as incorrectly detected S1 or S2 sounds, and a false negative (FN), as existing, but undetected S1 or S2 sounds. Finally the statistical parameter the accuracy (ACC) [3, 61] in percentages (%) was determined:
  $$\begin{array}{c} ACC=\frac{TP}{TP+FP+FN}\cdot 100. \end{array}$$ (1)
- *Signal-to-noise ratio improvement*—the parameter was set as the difference between the original SNR value of the disturbed signal (*SNR*_*in*_) and the SNR value of the filtered signal (*SNR*_*out*_). The higher the SNR improvement value, the more effective filtering was. The results are given in decibels (dB).
  $$\begin{array}{c} SNR_{in}=10{\text{log}}_{10}\frac{\sum_{m=1}^{M-1}{\left(fPCG_{ref}\left(m\right)\right)}^{2}}{\sum_{m=1}^{M-1}{\left(fPCG_{in}\left(m\right)-fPCG_{ref}\left(m\right)\right)}^{2}}, \end{array}$$ (2)
  $$\begin{array}{c} SNR_{out}=10{\text{log}}_{10}\frac{\sum_{m=1}^{M-1}{\left(fPCG_{ref}\left(m\right)\right)}^{2}}{\sum_{m=1}^{M-1}{\left(fPCG_{filt}\left(m\right)-fPCG_{ref}\left(m\right)\right)}^{2}}, \end{array}$$ (3)
  where *fPCG*_*ref*_(*m*) is the reference signal, *fPCG*_*in*_(*m*) is the input signal containing interference, *fPCG*_*filt*_(*m*) is the signal after application of the filtering method and *M* is the number of samples of the reference signal.
- *Mean error of heart interval measurement $\bar{|\Delta T_{i}|}$*—the parameter determines the mean value of the measurement error |Δ*T*_*i*_|, which was calculated as the absolute value of heart interval differences |Δ*T*_*i*_| in milliseconds (ms) [62]:
  $$\begin{array}{c} |\Delta T_{i}\left|=\right|T_{i_{filt}}-T_{i_{ref}}|, \end{array}$$ (4)
  where $T_{i_{filt}}$ is value i-of the interval of the filtered signal and $T_{i_{ref}}$ is value i-of the interval of the reference signal.

### Algorithms settings

In order to objectively test all filtering methods, it was necessary to find their optimal setting for each type and level of interference. That was achieved with the help of automated algorithm. For each combination of set parameters, the automated algorithm compared the filtered signal with the reference signal and calculated ACC values. The setting (as well as the filtered signal) with the highest ACC value was chosen. The whole process is shown in Fig 3.

**Fig 3:** Process of choosing the optimal setting of algorithm parameters.

For S-G filter, FIR filter, AWT and MODWT the optimal parameter settings are summarised in Table 2 and for VMD, EMD, EEMD and CEEMDAN in Table 3. For S-G filter it was necessary to set the length of the window and the polynomial order. For FIR filter it was necessary to choose an appropriate filter system (the BPF type with a frequency band of 20–110 Hz was used). For the AWT and MODWT methods it was necessary to choose an appropriate type of wavelet, wavelet width and number of decomposition levels. The *symlet*, *coiflet* and *Daubechies* wavelets were tested because their shape, energy and frequency spectrum is similar to that of fHSs [3]. For the EEMD a CEEMDAN methods it was necessary to choose the appropriate number of ensemble trials *N* and the standard deviation of the added noise *Nstd*. All four methods VMD, EMD, EEMD, and CEEMDAN were based on the principle of decomposition of the input signal into simpler signals-IMFs. The total number of extracted IMFs was dependent on the character of the input signal and extraction of IMFs took place as long as it was not possible to extract further IMFs. This was in the case where the signal was a constant, monotone function or a function with one extreme. For these methods it was therefore necessary to choose an appropriate combination of IMFs, which contributed to the creation of the resulting filtered signal. An example of three IMFs for the VMD, EMD, EEMD, and CEEMDAN methods is shown in Fig 4.

**Fig 4:** Example of three IMFs extracted by the a) VMD, b) EMD, c) EEMD, and d) CEEMDAN.

## Results

The efficiency of the S-G filter, FIR filter, AWT, MODWT, VMD, EMD, EEMD and CEEMDAN was evaluated against reference signals. In total 15 types of disturbance were filtered (four individual types of disturbance and eleven combinations) for two recordings r01 and r02. Evaluation of the effectiveness of the methods was carried out by detection of S1 and S2 sounds, calculation of SNR improvement and determination of parameter $\bar{|\Delta T_{i}|}$. The best result for the given type of disturbance was highlighted in the table (for detection of S1 and S2 sounds and SNR improvement the highest values were highlighted and for parameter $\bar{|\Delta T_{i}|}$ the lowest values).

### Accuracy of S1 and S2 sounds detection

Evaluation of the accuracy of S1 and S2 sounds detection was carried out by determining the values of TP, FP and FN, and then calculating the ACC parameter. The resulting ACC values for detection of S1 sounds for both recordings r01 and r02 are summarised in Table 4 and the resulting ACC values for detection of S2 sounds for both recordings r01 and r02 are summarised in Table 5.

According to Table 4 all tested algorithms, except VMD, achieved effective extraction and accurate detection of S1 sounds, as the average ACC values exceeded 80%. Based on the average of the ACC values, the most effective algorithm was the CEEMDAN (91.53%), followed by the EEMD method, which also achieved an average ACC value of over 90% (90.16%). The S-G filter, FIR filter, AWT, MODWT and EMD methods can be considered less suitable as their average ACC values did not exceed 90% (88.87%, 83.92%, 88.45%, 87.78%, and 84.92%, respectively). The VMD method reached an average accuracy of 78.84% and can be considered the least effective.

According to Table 5 in the detection of S2 sounds, lower accuracy was generally achieved, as none of the methods reached an average ACC value of over 80%. Based on the average of the ACC values, the most effective algorithm was the CEEMDAN (68.89%), followed by the MODWT (68.75%) and FIR filter (68.48%). The EEMD, EMD and S-G filter with an average accuracy of 66.50%, 63.36%, and 60.01%, respectively, can be considered even less effective. The S2 sounds were significantly suppressed by VMD and AWT, which reached the lowest average ACC values (52.10% and 49.34%, respectively).

### Signal-to-Noise ratio improvement

The resulting SNR improvement values are summarised for both recordings r01 and r02 in Table 6. The best results in SNR improvement were achieved with the CEEMDAN method with an average value of 9.75 dB, followed by EEMD with an average value of 8.30 dB. Lower average SNR improvement values were obtained by AWT (7.63 dB) and FIR filter (7.40 dB). These methods reached satisfactory results in some cases, but low in others which caused the average SNR improvement to be lower. For example, AWT achieved the highest SNR improvement in the case of Gaussian noise and ambient noise in both r01 and r02 recordings (14.10 dB, 11.23 dB, 13.96 dB, and 12.27 dB, respectively) or for the combination of Gaussian noise and ambient noise in r01 recording (12.08 dB). But on the other hand, in the case of mHSs in r02 recording, AWT achieved the lowest SNR improvement value (4.59 dB). The situation was similar for the FIR filter, which achieved the highest value of SNR improvement in the case of a combination of mHSs and Gaussian noise in r01 recording (11.91 dB) but the second lowest value in the case of a combination of movement artifacts, Gaussian and ambient noise in r02 recording (3.53 dB) or in the case of the combination of all four types of interference in r02 recording (3.31 dB). The lowest SNR improvement was achieved with VMD, S-G filter, EMD and MODWT (6.78 dB, 6.77 dB, 6.19 dB, and 5.60 dB, respectively).

### Mean error of heart interval measurement

The resulting values of the $\bar{|\Delta T_{i}|}$ parameter are summarised for both recordings r01 and r02 in Table 7. The lowest average $\bar{|\Delta T_{i}|}$ value and thus the best result was obtained again using the CEEMDAN method with an average value of 3.27 ms, followed by EEMD with an average value of 3.50 ms. Less effective were AWT, MODWT, S-G filter, VMD and EMD, as the average $\bar{|\Delta T_{i}|}$ values exceeded 4 ms (4.31 ms, 4.40 ms, 4.42 ms, 4.53 ms, and 4.78 ms, respectively). The FIR filter can be considered the least effective, as the average $\bar{|\Delta T_{i}|}$ value exceeded 5 ms (5.12 ms).

### Statistical analysis

To determine whether the differences of the results provided by the individual algorithms are statistically significant, we performed a statistical analysis of the results obtained for all evaluation parameters used (ACC when detecting S1 and S2, SNR improvement and $\bar{|\Delta T_{i}|}$). Statistical analysis was performed using *R Core Team* [63]. In all cases, statistical significance was set at p <0.05.

First, normality of the data was tested for each algorithm and each interference level using the Shapiro-Wilk test. In some cases, statistically significant deviations from normality were detected, and therefore non-parametric methods, median and interquartile range (IQR), were selected to describe the data. Descriptive statistics were performed separately for record r01, which was exposed to lower levels of interference (referred to as low noise level), and separately for record r02, which was subjected to higher levels of interference (referred to as high noise level).

The Kruskal-Wallis test was used to determine statistically significant differences between the compared algorithms in terms of individual evaluation parameters (*H*_0_: Medians of the evaluation parameter are the same for all algorithms, *H*_*A*_: Difference between at least one pair of medians of the evaluation parameters is statistically significant). If a statistically significant difference between the compared algorithms was detected for the medians of an evaluation parameter, a post hoc analysis was performed using Dunn’s test and multiple comparison p-values were adjusted with the Benjamin-Hochberg method.

For the ACC parameter, a statistically significant difference was found between the compared algorithms in the case of signals affected by low interference levels, both in the detection of S1 sounds and in the detection of S2 sounds (p-value <0.001 in both cases), see Table 8. In the case of S1 sounds detection, the VMD algorithm was identified as the algorithm with low ACC, the difference of the rest of the compared algorithms was not statistically significant in terms of the ACC parameter.

**Table 8:** Statistical analysis of ACC parameter depending on the compared algorithms.

Algorithms	ACC (%)			
	S1 sounds		S2 sounds	
	Low noise level Median (IQR)	High noise level Median (IQR)	Low noise level Median (IQR)	High noise level Median (IQR)
S-G	99.27 (96.17; 100.00)	80.67 (71.25; 91.85)	77.76 (64.23; 91.37)	36.16 (23.89; 57.83)
FIR	98.98 (91.35; 100.00)	72.94 (57.06; 94.83)	89.10 (78.69; 99.28)	42.42 (33.21; 75.74)
AWT	99.57 (97.44; 100.00)	85.55 (65.89; 93.22)	60.05 (52.95; 66.57)	32.61 (28.65; 46.34)
MODWT	99.57 (96.00; 100.00)	79.41 (63.28; 97.64)	86.25 (79.45; 95.27)	46.85 (38.48; 75.26)
VMD	88.46 (82.64; 88.64)	75.45 (61.22; 85.01)	65.95 (46.80; 75.97)	37.76 (26.61; 57.74)
EMD	98.70 (91.28; 100.00)	70.20 (61.65; 95.10)	87.19 (77.04; 95.92)	41.53 (25.59; 56.53)
EEMD	99.85 (98.62; 100.00)	91.51 (67.91; 97.49)	91.82 (72.27; 95.36)	45.21 (26.46; 64.44)
CEEMDAN	99.71 (95.50; 100.00)	92.49 (73.55; 97.84)	93.08 (82.76; 98.33)	36.98 (33.75; 77.07)
Between-groups diff. (p-value)	< 0.001^a^	0.355	< 0.001^b^	0.364

Kruskal-Wallis test for the between-group differences. Post-hoc analysis (homogenous subgroups):

^a^—(S-G, FIR, AWT, MODWT, EMD, EEMD, CEEMDAN), VMD,

^b^—(S-G, FIR, MODWT, EMD, EEMD, CEEMDAN), (S-G, AWT, VMD).

In the case of S2 sounds detection, two homogeneous subgroups of algorithms were identified, i.e. subgroups of algorithms where the difference between medians of the ACC parameter was not statistically significant. The first group consisted of the S-G, FIR, MODWT, EMD, EEMD, and CEEMDAN algorithms; the second homogeneous subgroup consisted of the S-G, AWT, and VMD algorithms. It can be noted that the S-G algorithm can be classified in terms of the ACC parameter both in the subgroup of algorithms with higher ACC and in the subgroup of algorithms with lower ACC.

For signal affected by high levels of interference, no statistically significant difference was observed between the compared algorithms in terms of ACC parameter in the detection of S1 sounds (p-value = 0.355), nor in the detection of S2 sounds (p-value = 0.364), see Table 8. A comparison of algorithms in S1 and S2 detection assessed by the ACC parameter is shown in Figs 5 and 6, respectively.

**Fig 5:** Hybrid boxplots providing comparison of the S1 detection assessed by ACC parameter for all compared algorithms and two interference levels (low and high).

**Fig 6:** Hybrid boxplots providing comparison of the S2 detection assessed by ACC parameter for all compared algorithms and two interference levels (low and high).

In the case of the SNR improvement, a statistically significant difference was found between the compared algorithms at low and high interference levels (in both cases p-value <0.001), see Table 9. At a low interference level, three homogeneous subgroups of algorithms were identified. The first two subgroups included algorithms with higher values of SNR improvement; the first subgroup consisted of FIR, AWT, EEMD, and CEEMDAN, the second subgroup consisted of S-G, FIR, AWT, VMD, and EMD. On the other hand, statistically significantly lowest values of SNR improvement were observed with the MODWT algorithm, forming the third subgroup. In the case of a high level of interference, the CEEMDAN algorithm was identified as the algorithm with the statistically significantly highest SNR improvement; no statistically significant differences were observed between the other algorithms.

**Table 9:** Statistical analysis of SNR improvement and $\bar{|\Delta T_{i}|}$ parameters depending on the compared algorithms.

Algorithms	SNR improvement (dB)		$\bar{|\Delta T_{i}|}$ (ms)	
	S1 sounds		S2 sounds	
	Low noise level Median (IQR)	High noise level Median (IQR)	Low noise level Median (IQR)	High noise level Median (IQR)
S-G	7.06 (6.08; 8.30)	5.98 (4.50; 7.49)	0.83 (0.24; 2.12)	7.19 (4.22; 10.91)
FIR	7.37 (6.87; 9.29)	6.19 (5.25; 8.05)	1.01 (0.16; 3.74)	9.34 (2.79; 12.45)
AWT	7.93 (6.14; 9.72)	6.04 (4.54; 8.22)	0.69 (0.22; 1.77)	6.44 (3.79; 11.50)
MODWT	4.67 (3.73; 5.08)	6.36 (5.62; 8.23)	0.76 (0.28; 2.33)	7.89 (1.73; 11.75)
VMD	6.78 (5.85; 6.96)	6.92 (6.03; 8.02)	0.83 (0.63; 3.48)	6.70 (2.92; 10.90)
EMD	7.33 (5.57; 9.11)	5.74 (3.40; 6.58)	1.15 (0.23; 3.49)	9.40 (2.27; 10.96)
EEMD	9.91 (8.73; 10.79)	7.80 (3.44; 9.49)	0.56 (0.14; 1.22)	4.56 (1.46; 9.80)
CEEMDAN	9.90 (8.02; 10.16)	9.74 (8.78; 10.95)	0.57 (0.22; 2.59)	3.91 (1.51; 9.84)
Between-groups diff. (p-value)	< 0.001^a^	< 0.001^b^	0.692	0.704

Kruskal-Wallis test for the between-group differences. Post-hoc analysis (homogenous subgroups):

^a^—(FIR, AWT, EEMD, CEEMDAN), (S-G, FIR, AWT, VMD, EMD), MODWT,

^b^—CEEMDAN, (S-G, FIR, AWT, MODWT, VMD, EMD, EEMD).

In the case of the parameter $\bar{|\Delta T_{i}|}$, no statistically significant difference was found between the compared algorithms, both for the signals affected by low interference levels (p-value = 0.692) and those affected with high interference levels (p-value = 0.704), see Table 9. Graphical presentation of the comparison of algorithms in terms of SNR improvement and $\bar{|\Delta T_{i}|}$ is demonstrated in Figs 7 and 8, respectively.

**Fig 7:** Hybrid boxplots providing comparison of the SNR improvement for all compared algorithms and two interference levels (low and high).

**Fig 8:** Hybrid boxplots providing comparison of the $\bar{|\Delta T_{i}|}$ for all compared algorithms and two interference levels (low and high).

To verify the effect of the interference level on the ACC parameter, the ACC ratios of the low and high interference levels for all compared algorithms were analyzed for both S1 and S2 sounds detection. Statistically significant difference (median ACC ratio less than or greater than one) meant that there was a statistically significant difference between ACC for low noise level and high noise level. The ACC ratio values greater than one thus indicated a higher ACC at low interference levels. Non-parametric methods were again used for descriptive statistics as well as for statistical induction methods. Significance of ACC ratio was tested by two-tailed Wilcoxon signed-rank test (*H*_0_: The median of ACC ratio is equal to one, *H*_*A*_: The median of ACC ratio is not equal to one). For all compared algorithms, both in the case of S1 sounds detection and in the case of S2 sounds detection, a statistically significant effect of the interference level on the ACC parameter was identified (in all cases p-values ≤ 0.002), see Table 10.

**Table 10:** Statistical analysis of ACC ratios (low noise level/high noise level) depending on the compared algorithms.

Algorithms	ACC ratio			
	S1 sounds		S2 sounds	
	Median (IQR)	Wilcoxon test (p-value)	Median (IQR)	Wilcoxon test (p-value)
S-G	1.23 (1.09; 1.35)	0.001	1.92 (1.56; 2.63)	<0.001
FIR	1.36 (1.05; 1.60)	0.001	1.78 (1.21; 2.10)	<0.001
AWT	1.16 (1.07; 1.48)	0.001	1.79 (1.57; 1.93)	<0.001
MODWT	1.25 (1.02; 1.52)	0.001	1.73 (1.26; 2.02)	<0.001
VMD	1.17 (1.04; 1.37)	<0.001	1.73 (1.17; 2.11)	<0.001
EMD	1.41 (1.05; 1.50)	<0.001	2.12 (1.64; 2.43)	<0.001
EEMD	1.09 (1.03; 1.45)	0.002	1.69 (1.47; 2.69)	<0.001
CEEMDAN	1.08 (1.02; 1.30)	0.001	1.83 (1.27; 2.43)	<0.001
Between-groups diff. (p-value)	0.725		0.579	

p-value of two-sided Wilcoxon signed-rank sum test: *H*_0_: The median of ACC ratio is equal to one.

Kruskal-Wallis test for the between-groups differences.

Finally, we used the Kruskal-Wallis test to find statistically significant differences between the compared algorithms with respect to the ACC ratio (*H*_0_: The medians of the ACC ratio are the same for all compared algorithms, *H*_*A*_: The difference of at least one pair of medians is statistically significant). With regard to the ACC ratio, no statistically significant difference was found between the compared algorithms, both in the detection of S1 sounds (p-value = 0.725) and in the detection of S2 sounds (p-value = 0.579), see Table 10. The Figs 9 and 10 provide a comparison of the algorithms using the hybrid boxplots in terms of the ACC ratio for S1 and S2 sounds, respectively.

**Fig 9:** Hybrid boxplots providing comparison of the ACC ratio (low noise level/high noise level) for S1 sounds detection.

**Fig 10:** Hybrid boxplots providing comparison of the ACC ratio (low noise level/high noise level) for S2 sounds detection.

## Discussion

Based on the evaluation of average values of objective parameters in the detection of S1 and S2 sounds, SNR improvement and $\bar{|\Delta T_{i}|}$ parameter, the best results were achieved using the CEEMDAN method. The EEMD method achieved very promising, although slightly worse results than CEEMDAN for all evaluated parameters. In addition, EEMD was computationally more complex than CEEMDAN. The EMD and VMD methods only achieved satisfactory results according to the parameter $\bar{|\Delta T_{i}|}$. In detection of S1 and S2 sounds and in SNR improvement its performance was poor. However, compared to the EEMD and CEEMDAN methods, their computational complexity was significantly lower. The AWT and MODWT methods achieved very promising results in detection of S1 sounds according to the $\bar{|\Delta T_{i}|}$ parameter. AWT achieved satisfactory results in SNR improvement, but on the other hand it achieved the worst average results of all methods in detection of S2 sounds. MODWT was effective in detection of S2 sounds, however it achieved the worst average results in SNR improvement. The FIR filter achieved satisfactory results in detection of S2 sounds and SNR improvement, however weak results in detection of S1 sounds and the worst results according to the $\bar{|\Delta T_{i}|}$ parameter. The S-G filter achieved very promising results in detection of S1 sounds and according to the $\bar{|\Delta T_{i}|}$ parameter, however in detection of S2 sounds and SNR improvement its performance was unsatisfactory.

In this section, the difference in extraction accuracy achieved by individual methods will be presented, especially in terms of S1 and S2 sounds detection. Furthermore, the influence of the interference level and the presence of multiple types of disturbance will be shown. An example of extracted signals for recording r02 loaded with individual types of disturbance is shown in Fig 11. It can be seen that all types of interference were sufficiently suppressed with regard to S1 sounds detection and S1 sounds could therefore be accurately detected (all methods in filtering of all four types of interference achieved ACC > 86%). However, during filtering mHSs, S-G filter, AWT, VMD and EMD were unable to effectively eliminate the maternal component, which led to lower accuracy in detection of S2 sounds (ACC < 81%). When filtering movement artifacts, elimination of interference was not sufficient using the S-G filter and AWT, which also led to very low accuracy in detection of S2 sounds (ACC < 60%). In the case of Gaussian noise, the AWT method effectively suppressed the interference, but in addition, the S2 sounds were also suppressed and their detection was therefore not successful (ACC = 60.81%). Detection of S2 sounds was also unsuccessful when using the VMD method, as interference was not sufficiently suppressed and S2 sounds were not correctly detected (ACC = 55.39%). When filtering ambient noise, the AWT and MODWT methods suppressed interference as well as S2 sounds, which led to low accuracy in their detection (ACC = 54.10% and 77.12%, respectively). On the other hand, the VMD and EMD methods were unable to sufficiently suppress interference and detection of S2 sounds was also inaccurate (ACC = 60.09% and 41.53%, respectively).

**Fig 11:** Comparison of extracted signals using all methods when filtering mHSs, movement artifacts, Gaussian noise, and ambient noise in recording r02.

The results of the study also showed the effect of level of interference on the resulting quality of the extracted signals, see Fig 12. Results for recording r01, which was loaded with a lower level of interference (SNR of signal with mHSs: -0.53 dB, movement artifacts: -0.84 dB, Gaussian noise: -1.20 dB, and ambient noise: -2.25 dB) were compared with recording r02, which was loaded with a higher level of interference (SNR of signal with mHSs: -1.82 dB, movement artifacts: -2.49 dB, Gaussian noise: -3.56 dB, and ambient noise: -5.74 dB). When filtering mHSs in recording r01 the maternal component was completely eliminated (in detection of S1 and S2 sounds ACC = 100%), however in the case of recording r02 residues of the maternal component remained in the signal. Although it did not significantly affect the accuracy of detection of S1 sounds (ACC = 99.13%), it decreased the accuracy of detection of S2 sounds (ACC = 92.89%). This was similar when filtering movement artifacts. In the case of recording r01 accurate detection of S1 (ACC = 100%) and S2 sounds (ACC = 98.41%) was achieved. But in the case of recording r02, the insufficient elimination of interference led to a fall in accuracy in detection of S1 sounds (ACC = 95.43%) and inaccurate detection of S2 sounds (ACC = 78.28%). When suppressing Gaussian noise, interference was effectively filtered in both recordings r01 and r02 and detection of S1 sounds was accurate (in both recordings ACC = 100%). However, residues of interference led to slightly worse extraction in recording r02 and lower accuracy in S2 sounds detection (ACC = 94.83%) compared to recording r01 (ACC = 99.27%). In the case of ambient noise, the level of interference also significantly influenced the resulting quality of the extracted signal. In recording r01 accurate detection of S1 (ACC = 100%) and S2 sounds (ACC = 98.7%) was achieved, but in the case of recording r02, interference was not filtered out, which led to less accurate detection of S1 (ACC = 97.69%) and S2 sounds (ACC = 84.58%).

**Fig 12:** Comparison of the resulting quality of the extracted signals by the CEEMDAN method depending on the level of interference.

As well as the level of interference, the presence of multiple types of disturbance influenced the overall extraction quality, see an example for recording r02 in Fig 13. If only mHSs were present in the signal, the interference was eliminated and accurate detection of S1 (ACC = 99.13%) and S2 sounds (ACC = 92.89%) was achieved. If movement artifacts were added to mHSs, residues of interference led to a slightly lower accuracy of S1 sounds detection (ACC = 95.53%), but a significantly lower accuracy of S2 sounds detection (ACC = 52.34%). When adding further interference in the form of Gaussian noise, the interference was not sufficiently suppressed. This led to significantly lower values of S1 (ACC = 80.23%) and S2 sounds (ACC = 34.64%) detection. The worst results in detection of S1 (ACC = 55.02%) and S2 sounds (ACC = 29.3%) was achieved when adding ambient noise, and therefore loading the signal with all four types of interference.

**Fig 13:** Comparison of presence of multiple types of disturbance on resulting quality of extracted signals using the CEEMDAN method.

## Summary and future directions

This study focused on the comparison of eight single-channel both conventional (S-G filter, FIR filter) and advanced (AWT, MODWT, VMD, EMD, EEMD, CEEMDAN) signal-processing algorithms. The use of a relatively large number of algorithms and objective evaluation parameters (accuracy of S1 and S2 sounds detection, SNR improvement and $\bar{|\Delta T_{i}|}$ parameter) can be considered as an advantage of this study. In particular, the evaluation of the accuracy of S2 detection is not very common in the field of fPCG (except for very few publications, e.g. [16–18]), although this information is useful for clinical practice. The benefit of the study is also to test the performance of algorithms in many scenarios, such as different types and levels of interference. Overall, the methods were tested on signals loaded with 30 levels of interference (SNR values from -0.53 dB to -10.76 dB), including the most common types of interference (mHSs, movement artifacts, Gaussian noise, ambient noise) and their combinations. In particular, testing on signals affected with more than one type of interference is valuable as it reflects situations that are very likely to occur when measuring in real conditions. In addition, to our best knowledge, some algorithms (MODWT or CEEMDAN) have not yet been tested and published at all for the fPCG extraction.

Conversely, performing experiments solely on synthetic signals can be considered a limitation of this study since tests on real signals can show slightly different results. In addition, testing was performed only on signals corresponding to the 40th week of pregnancy. As fPCG signals change throughout pregnancy, especially in terms of useful signal amplitude, further testing of algorithms on fPCG signals corresponding to other gestational ages is necessary. Another disadvantage may be offline testing, which may not fully address the problems associated with online implementation. This is associated mainly with the need to optimize algorithms in real time or to process the input signals piece-by-piece (as opposed to having the entire input signal available).

The results of statistical analysis presented herein showed no statistically significant difference between performance of the individual algorithms in terms of the parameter $\bar{|\Delta T_{i}|}$ at signals with low as well as high interference levels. For the ACC parameter, assessing the ability to detect S1 and S2, this applied at signals loaded by high interference levels. Contrary, when the signal was loaded with low levels of interference, a statistically significant difference was identified between the algorithms for the ACC parameter. A statistically significant difference between the algorithms was also found in the case of the SNR improvement parameter when the signal was loaded with both low and high levels of interference. Furthermore, for all compared algorithms, a statistically significant effect of the interference level on the ACC parameter was identified in the case of both S1 and S2 sounds detection. However, with respect to the ACC ratio (low noise level/high noise level), no statistically significant difference was found between the compared algorithms, both in the detection of S1 and S2.

Based on the evaluation of average values of objective parameters, CEEMDAN proved to be the most effective method for detecting S1 and S2 sounds with average accuracy of ACC = 91.53% in the detection of S1 and ACC = 68.89% when S2 is detected. In addition, CEEMDAN also outperformed the other tested methods in terms of improving SNR and the $\bar{|\Delta T_{i}|}$ parameter. Compared to EEMD, CEEMDAN was computationally faster and allowed implementation in real-time operating device. The benefits of the CEEMDAN algorithm can be summarized as follows:

- *Single-channel approach*—channel approach—provides higher comfort and mobility for the pregnant woman.
- *High quality extraction*—even for signals with relatively noisy signals.
- *High accuracy in detecting S1*—ensures the ability to determine fHR accurately.
- *Low computational complexity*—enables implementation in real-time operating devices.

On the other hand, accurate detection of S2 sounds proved to be difficult for all algorithms, including CEEMDAN. This was probably due to the lower magnitude of S2 compared to S1. As a result, S2 sounds were less distinct from noise and their subsequent extraction and detection was inaccurate. Therefore, future research should be focused on the refinement of S2 detection.

It would also be beneficial for clinical practice to detect and classify pathological heart murmurs that can help detect congenital heart defects. Algorithms based on artificial intelligence and machine learning could be used for classification of fetal pathological conditions. However, very few authors have dealt with the use of artificial intelligence and machine learning in the field of fPCG. This may be because these methods require a large amount of physiological and pathological data for both training and testing, but these data are not available in the field of fPCG. For these reasons, our further research will focus on creating a large dataset containing both real pathological and physiological fPCG records. The dataset will include information on fetal gestational age, sensor placement, maternal and fetal health, and reference annotations with fetal and maternal HSs locations will be created so that the efficiency of extraction algorithms can be objectively evaluated. Thus, other filtering methods will be further tested in the future, including multi-channel algorithms or hybrid methods combining multiple algorithms to achieve more accurate extraction.

## Conclusion

In this study eight algorithms were compared (S-G filter, FIR filter, AWT, MODWT, VMD, EMD, EEMD, and CEEMDAN) for fPCG extraction to eliminate mHSs, movement artifacts, Gaussian noise, ambient noise and eleven combinations of these disturbances. Testing was carried out on two synthetic recordings r01 and r02, where recording r02 was loaded with higher levels of interference than recording r01. The evaluation was performed by the assessment of the accuracy of S1 and S2 sounds detection, SNR improvement and $\bar{|\Delta T_{i}|}$ parameter. In all parameters the best results were achieved by the CEEMDAN method. Very promising results were also achieved using the EEMD method, however compared to CEEMDAN, EEMD was computationally more complex. It was shown that when loading an input signal with a higher level of interference or multiple types of disturbance, the quality of extraction was worsened and important clinical information was lost. When recording fPCG it is therefore necessary to ensure optimal conditions, particularly appropriate placing of the sensor and eliminating interference, which could unnecessarily contaminate a useful signal. Future research will focus on testing the CEEMDAN method on real physiological and pathological recordings and on creating our own database with real recordings which will be provided to the scientific community for testing extraction algorithms. Furthermore, other algorithms will be tested, including multichannel algorithms or hybrid methods combining multiple algorithms to increase extraction efficiency.

## References

[1] KovácsF, HorváthC,BaloghÁT, HosszúG. Fetal Phonocardiography—Past and Future Possibilities. Computer Methods and Programs in Biomedicine. 2011;104(1):19–25. doi: 10.1016/j.cmpb.2010.10.006 21146247

[2] HannaIR, SilvermanME. A History of Cardiac Auscultation and Some of Its Contributors. The American Journal of Cardiology. 2002;90(3):259–267. doi: 10.1016/S0002-9149(02)02465-7 12173582

[3] MartinekR, BarnovaK, JarosR, KahankovaR, KupkaT, JezewskiM, et al. Passive Fetal Monitoring by Advanced Signal Processing Methods in Fetal Phonocardiography. IEEE Access. 2020;8:221942–221962. doi: 10.1109/ACCESS.2020.3043496

[4] Chetlur AdithyaP, SankarR, MorenoWA, HartS. Trends in Fetal Monitoring through Phonocardiography: Challenges and Future Directions. Biomedical Signal Processing and Control. 2017;33:289–305. doi: 10.1016/j.bspc.2016.11.007

[5] CesarelliM, RuffoM, RomanoM, BifulcoP. Simulation of Foetal Phonocardiographic Recordings for Testing of FHR Extraction Algorithms. Computer Methods and Programs in Biomedicine. 2012;107(3):513–523. doi: 10.1016/j.cmpb.2011.11.008 22178069

[6] GangulyA, SharmaM. Detection of Pathological Heart Murmurs by Feature Extraction of Phonocardiogram Signals. Journal of Applied and Advanced Research. 2017; p. 200–205. doi: 10.21839/jaar.2017.v2i4.94

[7] KovácsF, KersnerN, KádárK, HosszúG. Computer Method for Perinatal Screening of Cardiac Murmur Using Fetal Phonocardiography. Computers in Biology and Medicine. 2009;39(12):1130–1136. doi: 10.1016/j.compbiomed.2009.10.001 19897185

[8] BaloghAT. Analysis of the Heart Sounds and Murmurs of Fetuses and Preterm Infants. Pazmany Peter Katolikus Egyetem; 2015.

[9] ChourasiaJ, ChourasiaV, MittraAK. Prenatal Detection of Congenital Heart Defects: Study & Comparative Analysis of Existing Techniques. International Journal. 2017;5(2).

[10] IbrahimEA, Al AwarS, BalayahZH, HadjileontiadisLJ, KhandokerAH. A Comparative Study on Fetal Heart Rates Estimated from Fetal Phonography and Cardiotocography. Frontiers in Physiology. 2017;8:764. doi: 10.3389/fphys.2017.00764 29089896PMC5651042

[11] MondalH, MondalS, SahaK. Development of a Low-Cost Wireless Phonocardiograph With a Bluetooth Headset under Resource-Limited Conditions. Medical Sciences. 2018;6(4):117. doi: 10.3390/medsci6040117 30563004PMC6313612

[12] KovácsF, TörökM, HorváthC, BaloghÁT, ZsedrovitsT, NagyA, et al. A New, Phonocardiography-Based Telemetric Fetal Home Monitoring System. Telemedicine and e-Health. 2010;16(8):878–882. doi: 10.1089/tmj.2010.0039 20925563

[13] Sbrollini A, Strazza A, Caragiuli M, Mozzoni C, Tomassini S, Agostinelli A, et al. Fetal Phonocardiogram Denoising by Wavelet Transformation: Robustness to Noise. In: 2017 Computing in Cardiology Conference; 2017.

[14] VadaliVABK. A Comparative Study of Signal Processing Methods for Fetal Phonocardiography Analysis. University of South Florida; 2018.

[15] TomassiniS, StrazzaA, SbrolliniA, MarcantoniI, MorettiniM, FiorettiS, et al. Wavelet Filtering of Fetal Phonocardiography: A Comparative Analysis. Mathematical Biosciences and Engineering. 2019;16(5):6034–6046. doi: 10.3934/mbe.2019302 31499751

[16] MittraAK, ChoudhariNK. Time-frequency analysis of foetal heart sound signal for the prediction of prenatal anomalies. Journal of Medical Engineering & Technology. 2009-07-09;33(4):296–302. doi: 10.1080/03091900802454384 19384705

[17] KoutsianaE, HadjileontiadisLJ, ChouvardaI, KhandokerAH. Fetal Heart Sounds Detection Using Wavelet Transform and Fractal Dimension. Frontiers in Bioengineering and Biotechnology. 2017;5:49. doi: 10.3389/fbioe.2017.00049 28944222PMC5596097

[18] VaismanS, Yaniv SalemS, HolcbergG, GevaAB. Passive Fetal Monitoring by Adaptive Wavelet Denoising Method. Computers in Biology and Medicine. 2012;42(2):171–179. doi: 10.1016/j.compbiomed.2011.11.005 22169397

[19] ChourasiaVS, TiwariAK. Design Methodology of a New Wavelet Basis Function for Fetal Phonocardiographic Signals. The Scientific World Journal. 2013;2013:1–12. doi: 10.1155/2013/505840 23766693PMC3676936

[20] Jiménez-GonzálezA, JamesCJ. Extracting Sources from Noisy Abdominal Phonograms: A Single-Channel Blind Source Separation Method. Medical & Biological Engineering & Computing. 2009;47(6):655–664. doi: 10.1007/s11517-009-0474-8 19301051

[21] Warbhe AD, Dharaskar RV, Kalambhe B. A Single Channel Phonocardiograph Processing Using EMD, SVD, and EFICA. In: 2010 3rd International Conference on Emerging Trends in Engineering and Technology. Goa: IEEE; 2010. p. 578–581.

[22] Samieinasab M, Sameni R. Fetal Phonocardiogram Extraction Using Single Channel Blind Source Separation. In: 2015 23rd Iranian Conference on Electrical Engineering. Tehran, Iran: IEEE; 2015. p. 78–83.

[23] KovacsF, HorváthC,BaloghÁT, HosszúG. Extended Noninvasive Fetal Monitoring by Detailed Analysis of Data Measured With Phonocardiography. IEEE Transactions on Biomedical Engineering. 2011;58(1):64–70. doi: 10.1109/TBME.2010.2071871 20813630

[24] RuffoM, CesarelliM, RomanoM, BifulcoP, FratiniA. An Algorithm for FHR Estimation from Foetal Phonocardiographic Signals. Biomedical Signal Processing and Control. 2010;5(2):131–141. doi: 10.1016/j.bspc.2010.02.002

[25] Soysa WNM, Godaliyadda RI, Wijayakulasooriya JV, Ekanayake MPB, Kandauda IC. Extraction and Analysis of Fetal Heart Signals with Abnormalities an Eigen-analysis Based Approach. In: 2013 IEEE 8th International Conference on Industrial and Information Systems. Peradeniya, Sri Lanka: IEEE; 2013. p. 294–299.

[26] Dia N, Fontecave-Jallon J, Gumery PY, Rivet B. Fetal Heart Rate Estimation from a Single Phonocardiogram Signal Using Non-Negative Matrix Factorization. In: 2019 41st Annual International Conference of the IEEE Engineering in Medicine and Biology Society (EMBC). Berlin, Germany: IEEE; 2019. p. 5983–5986.10.1109/EMBC.2019.885722031947210

[27] HuiminW, XingyuL. Extraction Method of Fetal Phonocardiogram Based on Lifting Wavelet Analysis. Journal of Physics: Conference Series. 2020;1544(1):012103.

[28] ZahorianSA, ZuckerwarAJ, KarnjanadechaM. Dual Transmission Model and Related Spectral Content of the Fetal Heart Sounds. Computer Methods and Programs in Biomedicine. 2012;108(1):20–27. doi: 10.1016/j.cmpb.2011.12.006 22285458

[29] DaiW, SelesnickI, RizzoJR, RuckerJ, HudsonT. A Nonlinear Generalization of the Savitzky-Golay Filter and the Quantitative Analysis of Saccades. Journal of Vision. 2017;17(9):10. doi: 10.1167/17.9.10 28813566PMC5852949

[30] OstertagovaE, OstertagO. Methodology and Application of Savitzky-Golay Moving Average Polynomial Smoother. Global J Pure Applied Math. 2016;12:3201–3210.

[31] OrfanidisSJ. Introduction to Signal Processing. Pearson Education, Inc; 2016.

[32] ZhdanovDS, BureevAS, KutsovMS, KiselevaEY, KistenevYV. Algorithm for Extraction of Fetal Heart Tones during Fetal Phonocardiography. Biol Med (Aligarh). 2015;7(3):2.

[33] WuJMT, TsaiMH, HuangYZ, IslamSH, HassanMM, AlelaiwiA, et al. Applying an Ensemble Convolutional Neural Network with Savitzky–Golay Filter to Construct a Phonocardiogram Prediction Model. Applied Soft Computing. 2019;78:29–40. doi: 10.1016/j.asoc.2019.01.019

[34] KrishnanPT, BalasubramanianP, UmapathyS. Automated Heart Sound Classification System from Unsegmented Phonocardiogram (PCG) Using Deep Neural Network. Physical and Engineering Sciences in Medicine. 2020;43(2):505–515. doi: 10.1007/s13246-020-00851-w 32524434

[35] Marchon N. Efficient FIR Filters for Biomedical Signals. In: TENCON 2019—2019 IEEE Region 10 Conference (TENCON). Kochi, India: IEEE; 2019. p. 1947–1951.

[36] WulfM, StaudeG, KnoppA, FelderhoffT. Efficient Design of FIR Filter Based Low-Pass Differentiators for Biomedical Signal Processing. Current Directions in Biomedical Engineering. 2016;2(1):215–219. doi: 10.1515/cdbme-2016-0048

[37] CherifLH, MostafiM, DebbalSM. Digital Filters in Heart Sound Analysis. International Journal of Clinical Medicine Research. 2014;1(3):97–108.

[38] RafieeJ, RafieeMA, PrauseN, SchoenMP. Wavelet Basis Functions in Biomedical Signal Processing. Expert Systems with Applications. 2011;38(5):6190–6201. doi: 10.1016/j.eswa.2010.11.050

[39] Alarcon-AquinoV, BarriaJA. Change Detection in Time Series Using the Maximal Overlap Discrete Wavelet Transform. Latin American applied research. 2009;39(2):145–152.

[40] StarckJL, FadiliJ, MurtaghF. The Undecimated Wavelet Decomposition and Its Reconstruction. IEEE Transactions on Image Processing. 2007;16(2):297–309. doi: 10.1109/TIP.2006.887733 17269625

[41] AlkhodariM, FraiwanL. Convolutional and Recurrent Neural Networks for the Detection of Valvular Heart Diseases in Phonocardiogram Recordings. Computer Methods and Programs in Biomedicine. 2021;200:105940. doi: 10.1016/j.cmpb.2021.105940 33494031

[42] DragomiretskiyK, ZossoD. Variational Mode Decomposition. IEEE Transactions on Signal Processing. 2014;62(3):531–544. doi: 10.1109/TSP.2013.2288675

[43] IshamMF, LeongMS, LimMH, AhmadZA. Variational Mode Decomposition: Mode Determination Method for Rotating Machinery Diagnosis. Journal of Vibroengineering. 2018;20(7):2604–2621. doi: 10.21595/jve.2018.19479

[44] Sujadevi VG, Soman KP, Kumar SS, Mohan N, Arunjith AS. Denoising of Phonocardiogram Signals Using Variational Mode Decomposition. In: 2017 International Conference on Advances in Computing, Communications and Informatics (ICACCI). Udupi: IEEE; 2017. p. 1443–1446.

[45] Nie Z. A Fetal Heart Sound Signal De-Noising Approach Based on VMD and JADE Algorithm. In: Proceedings of the 2018 International Conference on Network, Communication, Computer Engineering (NCCE 2018). Chongqing, China: Atlantis Press; 2018.

[46] GeH, ChenG, YuH, ChenH, AnF. Theoretical Analysis of Empirical Mode Decomposition. Symmetry. 2018;10(11):623. doi: 10.3390/sym10110623

[47] Attoh-OkineN, BarnerK, BentilD, ZhangR. The Empirical Mode Decomposition and the Hilbert-Huang Transform. EURASIP Journal on Advances in Signal Processing. 2008;2008(1):251518, 2008/251518. doi: 10.1155/2008/251518

[48] LinJ. Improved Ensemble Empirical Mode Decomposition Method and Its Simulation. In: LeeG, editor. Advances in Intelligent Systems. vol. 138. Berlin, Heidelberg: Springer Berlin Heidelberg; 2012. p. 109–115.

[49] IsmailS, SiddiqiI, AkramU. Localization and Classification of Heart Beats in Phonocardiography Signals —a Comprehensive Review. EURASIP Journal on Advances in Signal Processing. 2018;2018(1):26. doi: 10.1186/s13634-018-0545-9

[50] CheemaA, SinghM. An Application of Phonocardiography Signals for Psychological Stress Detection Using Non-Linear Entropy Based Features in Empirical Mode Decomposition Domain. Applied Soft Computing. 2019;77:24–33. doi: 10.1016/j.asoc.2019.01.006

[51] GhoshPK, PooniaD. Comparison of Some EMD Based Technique for Baseline Wander Correction in Fetal ECG Signa. International Journal of Computer Applications. 2015;116(15):48–52. doi: 10.5120/20416-2836

[52] WuZ, HuangNE. Ensemble Empirical Mode Decomposition: A Noise-assisted Data Analysis Method. Advances in Adaptive Data Analysis. 2009;01(01):1–41. doi: 10.1142/S1793536909000047

[53] PapadaniilCD, HadjileontiadisLJ. Efficient Heart Sound Segmentation and Extraction Using Ensemble Empirical Mode Decomposition and Kurtosis Features. IEEE Journal of Biomedical and Health Informatics. 2014;18(4):1138–1152. doi: 10.1109/JBHI.2013.2294399 25014929

[54] JimenezJA, BecerraMA, Delgado-TrejosE. Heart Murmur Detection Using Ensemble Empirical Mode Decomposition and Derivations of the Mel-Frequency Cepstral Coefficients on 4-Area Phonocardiographic Signals. In: Computing in Cardiology 2014. IEEE; 2014. p. 493–496.

[55] ColominasMA, SchlotthauerG, TorresME. Improved Complete Ensemble EMD: A Suitable Tool for Biomedical Signal Processing. Biomedical Signal Processing and Control. 2014;14:19–29. doi: 10.1016/j.bspc.2014.06.009

[56] LiuT, LuoZ, HuangJ, YanS. A Comparative Study of Four Kinds of Adaptive Decomposition Algorithms and Their Applications. Sensors. 2018;18(7):2120. doi: 10.3390/s18072120 30004429PMC6068995

[57] ChengX, WangP, SheC. Biometric Identification Method for Heart Sound Based on Multimodal Multiscale Dispersion Entropy. Entropy. 2020;22(2):238. doi: 10.3390/e22020238 33286012PMC7516671

[58] Tu Z, Cao G, Li Q, Xianxia Zhang, Jun Shi. Improved Methods for Detecting Main Components of Heart Sounds. In: 2010 Sixth International Conference on Natural Computation. Yantai, China: IEEE; 2010. p. 3585–3588.

[59] GoldbergerAL, AmaralLAN, GlassL, HausdorffJM, IvanovPC, MarkRG, et al. PhysioBank, PhysioToolkit, and PhysioNet: Components of a New Research Resource for Complex Physiologic Signals. Circulation. 2000;101(23). doi: 10.1161/01.CIR.101.23.e215 10851218

[60] BarnovaK, KahankovaR, JarosR, MartinekR. Synthetic Abdominal PCG Signals and Extracted Fetal PCG Signals. 2022.

[61] BilleciL, VaraniniM. A Combined Independent Source Separation and Quality Index Optimization Method for Fetal ECG Extraction from Abdominal Maternal Leads. Sensors. 2017;17(5):1135. doi: 10.3390/s17051135 28509860PMC5470811

[62] KupkaT, MatoniaA, JezewskiM, JezewskiJ, HorobaK, WrobelJ, et al. New Method for Beat-to-Beat Fetal Heart Rate Measurement Using Doppler Ultrasound Signal. Sensors. 2020;20(15):4079. doi: 10.3390/s20154079 32707863PMC7435740

[63] R: The R Project for Statistical Computing;. https://www.r-project.org/.

